The article "In Vitro Evaluation of Cytotoxic Potential of Caladium lindenii Extracts on Human Hepatocarcinoma HepG2 and Normal HEK293T Cell Lines" was retracted in 2023. Reasons: signs of a paper mill; suspected computer-generated content; unreliable results or conclusions; concerns about the data.

# *In Vitro* Evaluation of Cytotoxic Potential of *Caladium lindenii* Extracts on Human Hepatocarcinoma HepG2 and Normal HEK293T Cell Lines

**DOI:** 10.1155/2022/1279961

**Published:** 2022-09-22

**Authors:** Aasia Kalsoom, Awais Altaf, Muhammad Ashraf, Muhammad Muddassir Ali, Saira Aftab, Huma Sattar, Muhammad Sajjad, Amjad Islam Aqib, Tahir Maqbool

**Affiliations:** ^1^Institute of Molecular Biology and Biotechnology, The University of Lahore, Lahore 54000, Pakistan; ^2^Institute of Biochemistry and Biotechnology, University of Veterinary and Animal Sciences, Lahore 54000, Pakistan; ^3^Postdoctoral Fellow Department of Biochemistry and Biophysics, Stockholm University, Stockholm A 425-B16, Sweden; ^4^School of Biological Sciences, University of the Punjab, Lahore 54000, Pakistan; ^5^Department of Medicine, Cholistan University of Veterinary and Animal Sciences, Bahawalpur 63100, Pakistan

## Abstract

Data regarding the therapeutic potential of *Caladium lindenii* (*C. lindenii*) are insufficient. It becomes more important to explore plants as an alternative or palliative therapeutics in deadly diseases around the globe. The current study was planned to explore *C. lindenii* for its anticancer activity of ethanolic and hexane extracts of *C. lindenii* leaves against hepatic carcinoma (HepG2) and human embryonic kidney (HEK293T) cell lines. HepG2 and HEK293T cells were treated with 10, 50, 100, 200, and 400 *μ*g/mL of ethanolic and hexane extracts of *C. lindenii* and were incubated for 72 h. Antiproliferative activity was measured by 3-(4,5-dimethylthiazol-2yl)-2,5-biphenyl tetrazolium bromide (MTT) assay, and percentage viability were calculated through crystal violet staining and cellular morphology by Floid Cell Imaging Station. The study showed ethanolic extract exhibiting a significantly higher antiproliferative effect on HepG2 (IC50 = 31*μ*g/mL) in a concentration-dependent manner, while HEK293T (IC50 = 241*μ*g/mL) cells showed no toxicity. Hexane extract exhibited lower cytotoxicity (IC50 = 150*μ*g/mL) on HepG2 cells with no effect on HEK293T (IC50 = 550*μ*g/mL). On the other hand, the percentage viability of HepG2 cells was recorded as 78%, 67%, 50%, 37%, and 28% by ethanolic extracts, and 88%, 80%, 69%, 59%, and 50% by hexane extracts at tested concentrations of both extracts. Toxicity assay showed significantly safer ranges of percentage viabilities in normal cells (HEK293T), i.e., 95%, 90%, 88%, 76%, and 61% with ethanolic extract and 97%, 95%, 88%, 75%, and 62% with hexane extract. The assay validity revealed 100% viability in the control negative (dimethyl sulfoxide treated) and less than 45% in the control positive (cisplatin) on both HepG2 and HEK293T cells. Morphological studies showed alterations in HepG2 cells upon exposure to >50 *μ*g/mL of ethanolic extracts and ≥400 *μ*g/mL of hexane extracts. HEK293T on the other hand did not change its morphology against any of the extracts compared to the aggressive changes on the HepG2 cell line by both extracts and positive control (cisplatin). In conclusion, extracts of *C. lindenii* are proved to have significant potential for cytotoxicity-induced apoptosis in human cancer HepG2 cells and are less toxic to normal HEK293T cells. Hence *C. lindenii* extracts are proposed to be used against hepatocellular carcinoma (HCC) after further validations.

The article "In Vitro Evaluation of Cytotoxic Potential of Caladium lindenii Extracts on Human Hepatocarcinoma HepG2 and Normal HEK293T Cell Lines" was retracted in 2023. Reasons: signs of a paper mill; suspected computer-generated content; unreliable results or conclusions; concerns about the data.

## 1. Introduction

Due to the critical premise of epidemiology, cancer assures the most complex pathological state among the health of the population [1]. In 2018, 18 million people were affected by cancer including 8.5 million females and 9.5 million males from which 9.5 million deaths were reported. Approximately, 19.3 million new cancer cases and 10.0 million deaths have been reported in 2020. The estimation of cancer incidence is expected to be 28.4 million cases by the year 2040 [2]. Conventional medicines stimulate apoptosis and exploit the cascade of intracellular events in cancer cells. In the earliest times, various natural remedies had been used to manage diseases counting cancer, as these products have diversified mechanisms comprising the onset of apoptosis to inhibit signaling [3]. Morphological, biochemical, and gene-based characterization of cell lines come up with new intuitions regarding the diversity of polygenic traits, chemotherapy resistance, and the understanding of targeted cancer therapies [4].

Plant-based phytochemicals and antioxidants are known for anticancer treatment because of their anti-\proliferative, antioxidative, and apoptotic values in recent times [5]. Polyphenols are a large family of naturally occurring compounds with antioxidant properties. Volatile organic compounds (VOC) are responsible for aromatic characteristics in medicinal and aromatic plants (MAPs). These polyphenols can combat various diseases including neurodegenerative diseases, cardiovascular diseases, inflammations, and different types of cancers. The two existing biosynthetic pathways of secondary metabolites which lead to the formation of phenolic compounds are the shikimic acid pathway gives rise to phenylpropanoids, tannins, lignin, and many others, while the acetate-mevalonate pathway produces phenols [6]. Vegetables and MAPs are enriched with phenolic compounds (isoflavonoids, anthocyanins, lignans, and phenols). Their therapeutic effects on human health have been studied more efficiently in recent years. Flavonoids belong to the group of polyphenolic secondary metabolites found in plants and vegetables are responsible for health benefits through signaling pathways and antioxidant effects [7].

The article "In Vitro Evaluation of Cytotoxic Potential of Caladium lindenii Extracts on Human Hepatocarcinoma HepG2 and Normal HEK293T Cell Lines" was retracted in 2023. Reasons: signs of a paper mill; suspected computer-generated content; unreliable results or conclusions; concerns about the data.

The enormous therapeutic nature of medicinal plants are phytocompounds that provide a revolutionary advantage everywhere on the globe due to their hidden epitome [8]. A lot of analgesics, narcotics, and other drugs have been used since ancient times including opium, aspirin, quinine, and digitalis. Identified phytocompounds recommended for cancer treatment are vinca alkaloids, podophyllotoxin, taxanes, and roscovitine, and their derivatives have considerable effects on cancer development and proliferation. Because of diverse ethnomedicinal and ethnopharmacological comparisons of various species, many scientific works have been assembled over the past decade. Many phytocompounds including gingerol, curcumin, kaemferol, resveratrol, and nutritional phenolic compounds revealed anticancer activity both *in vivo* and *in vitro* experimentation [9]. Many *in vivo* as well as *in vitro* studies have reported the anticancerous properties of plant-derived natural compounds through the inhibition of enzymatic activity, stimulating DNA repair pathways, bringing antioxidant mechanism, and the release of protective enzymes [10].

*C. lindenii* is a flowering plant native to South America and belongs to the family Araceae. Many species of *Caladium* grow in wild areas of Nigeria. Authors reported that the plant parts of *Caladium* species have been used to manage various disease conditions including various kinds of tumors and infections in traditional medicine system [11]. The leaves, tubers, and other parts of *C. lindenii* were used therapeutically for stingray lesions in the regions of Brazil. However, no sufficient data has been found to reveal the presence of phytochemicals and pharmacological effects of *C. lindenii* in literature [12]. The underlying principle of the current research work is to explore the efficacy of organic extracts of *C. lindenii* with antiproliferative activity in response to the HepG2 (liver cancer) and normal HEK293T (human embryonic kidney 293T) cell lines.

## 2. Materials and Methods

### 2.1. Plant Collection and Identification

The leaves of *C. lindenii* were collected in the summer season from the botanical garden of Quaid-e-Azam University, Islamabad, Pakistan. The identification of leaves was confirmed by taxonomist Dr. Zaheer-ud-Din Khan (GC. Herb. Bot. 3854) working as a legendary professor in the Department of Botany, Government College University Lahore, and the samples were also submitted at the University Herbarium bank.

The article "In Vitro Evaluation of Cytotoxic Potential of Caladium lindenii Extracts on Human Hepatocarcinoma HepG2 and Normal HEK293T Cell Lines" was retracted in 2023. Reasons: signs of a paper mill; suspected computer-generated content; unreliable results or conclusions; concerns about the data.

### 2.2. Plant Extract Preparation

The leaves of *C. lindenii* were shade dried for 10 days and then crushed into the powdered form using a laboratory grinding mill (Thomas Scientific). Powdered leaves (300 g) were macerated into 1.0 L of ethanol (Sigma-Aldrich, 90%) and *n*-hexane (Sigma-Aldrich, 95%) separately and incubated for 2 weeks at 37°C. Filtration was done by using Whatman No.1 filter paper in reagent bottles. A rotary evaporator (Heidolph Hei-Vap, Germany) was used to concentrate the filtrates separately under a vacuum at 40°C, and the lyophilization or freeze-drying method was used to achieve dry extracts, and then samples were stored at 4°C [13].

### 2.3. Cancer Cell Cultivation

Hepatocellular carcinoma (HepG2) cell line and the human embryonic kidney (HEK293T) cell line were arranged from the UOL cell line BioBank (IMBB/CRiMM), The University of Lahore, Lahore, Pakistan. The cancer cells were successfully cultured in Dulbecco's Modified Eagle's Medium (DMEM) (Caisson Lot#02160032), 10% heat-inactivated fetal bovine serum (FBS) (Sigma-Aldrich Lot#BCBS3184V), and 100 U/mL of *Penicillin-Streptomycin* (Caisson Lot#10201011). The normal human kidney cells (HEK293T) were grown in Minimum Essential Media (MEM) (Gibco) with 15% FBS and incubated at 37°C with 5% CO_2_. Once the cells reach 80% confluent, the passage was carried out with minor changes. The medium was then removed and the cells were washed with PBS (Inovatiqa Lot#153595). Trypsinization was done by adding 3 mL of trypsin (Gibco Lot#1297823) until cells detach from the surface of the flask. A complete medium (5 mL) was added to end up the reaction, centrifuged the cells at 1500 rpm for 5 minutes, and then aspirated the supernatant. The passage was carried out by adding 10 mL of fresh growth medium and every 5 mL of cell suspension was shifted to a T75 cm^2^ cell culture flask [14].

### 2.4. Cell Counting and MTT Assay for Cytotoxicity Analysis

Trypsin was applied to cells to detach from the surface. Centrifugation was carried out and the cells were resuspended in 3 mL of the active medium. The hemocytometer was used for cell counting. The cell suspension was then placed into 96-well microtitre plastic plates and incubated at 37°C for 24 h with 5% CO_2_. The MTT assay was performed with slight modifications following the protocol described by Riaz [15]. The ethanolic and hexane crude extracts of *C. lindenii* were dissolved in dimethyl sulfoxide (DMSO) (Invitrogen Inc., USA) at a concentration of 160 mg/mL. HepG2 cells were seeded in 96-well microtitre plate (1 × 10^4^ cells/well) in 200 *μ*L of the complete medium in the microtitre plate, and the prepared concentrations (400, 200, 100, 50, and, 10 *μ*g/mL) were administered to cells. The last step was to incubate under the temperature mentioned previously with 5% CO_2_. The same protocol was used for HEK239T cells with MEM medium and 15% of FBS. Cisplatin drug (Patients Welfare Society Inmol Receipt No, 651278) (10 *μ*g/mL) was used as a positive control, DMSO (0.1%) as a negative control, and untreated cells containing plan DMEM medium (2% FBS) were used for the comparison, before and after treatment. The normal HEK293T and cancer HepG2 cell lines were used to assess the toxicity of plant extracts on healthy and cancer cells. After 72 h of incubation, the medium aspired and the degree of cellular proliferation was observed under the microscope. MTT assay was performed by adding 20 *μ*L of MTT reagent (Invitrogen Inc., USA) into each well and continued with incubation for 2 h. After removing the supernatant, 150 *μ*L of DMSO was mixed and then placed on a plate shaker to dissolve formazan crystals. After incubation for 15 minutes, the absorption spectra across the wells were determined by using a microplate reader (BIO-RAD) at a specified wavelength of 570 nm. Reactions in triplicate were performed for all samples. Half-maximal inhibitory concentration IC50 was calculated using a linear regression method.

The article "In Vitro Evaluation of Cytotoxic Potential of Caladium lindenii Extracts on Human Hepatocarcinoma HepG2 and Normal HEK293T Cell Lines" was retracted in 2023. Reasons: signs of a paper mill; suspected computer-generated content; unreliable results or conclusions; concerns about the data.

### 2.5. Cell Viability/Adhesion Assay

Crystal violet solution (0.1% wv) (Sigma-Aldrich) was prepared in 9 mL of PBS. Crystal violet (CV) assay was performed by following the protocol of Nawaz et al. with slight changes [16]. HepG2 and HEK293T cells were seeded in a 96-well microtitre plate (1 × 10^4^ cells/well) in 200 *μ*L of complete medium. Incubation was carried out for 72 h under a specified temperature (37°C) with humidity and 5% CO_2_. The treated (with plant extract) and untreated media were removed, and the cells were fixed with 70% ethanol for 10 min. CV solution was added for cell staining and stayed for 30 min. The plate was washed with PBS and then destained the cells with 200 *μ*L of triton X-100 solution (Sigma-Aldrich CAS#9036-19-5) used to de-stain cells. The cells were incubated at room temperature for 30 min and the optical density (OD) of samples was measured in triplicate at 570 nm using a spectrophotometer.

### 2.6. Percentage Calculation of Cell Viability

The percentage of viable cells was calculated by using the formula equation:

(1) $$\begin{array}{c} \%\text{Cell viability}=\frac{\text{Mean absorbance of treated cells}}{\text{Mean absorbance of control}}*100. \end{array}$$

### 2.7. Morphological Examination

To inspect the effect of plant extracts on cancer cell proliferation, the morphological variations were visualized and compared with the control group by applying different treatment concentrations on HepG2 and HEK293T cells using Floid Cell Imaging Station.

The article "In Vitro Evaluation of Cytotoxic Potential of Caladium lindenii Extracts on Human Hepatocarcinoma HepG2 and Normal HEK293T Cell Lines" was retracted in 2023. Reasons: signs of a paper mill; suspected computer-generated content; unreliable results or conclusions; concerns about the data.

### 2.8. Data Analysis

The experiments were carried out in three corresponding or identical parts and the data were expressed as mean ± standard deviation (SD). One-way analysis of variance (ANOVA) and Tukey's test were used to determine the interaction among three variables through Graph pad prism 5.0. IC50 values were calculated by linear regression method using AA Bioquest calculator. *p*˂0.05 was considered statistically significant with a confidence interval (CI) of 95%.

## 3. Results

### 3.1. Cytotoxic Effects of Plant Extracts on HepG2 and HEK-293T Cells

Cell proliferation inhibition activity of ethanol and hexane extracts of *C. lindenii* leaves on HepG2 and HEK-293 cell lines are represented in Figure 1 and Table 1. Depending on the results, the MTT test on the ethanolic extract showed a high antiproliferative effect against HepG2 (IC50 = 31*μ*g/mL) in comparison with HEK293T (IC50 = 241*μ*g/mL) at 72 h. It confounds that ethanolic extract concentrations (400, 200, 100, 50, 10 *μ*g/mL) become more toxic to cancer cells as compared to cisplatin (10 *μ*g/mL) which was taken as positive control and DMSO as negative control (Figure 1). Hence, the ethanolic extract enhanced the mortality of cancer cells even at the lowest concentration (50 *μ*g/mL). The wells treated with hexane extract exhibited lower cytotoxicity (IC50 = 150*μ*g/mL) on HepG2 cells, however, HEK293T (IC50 = 550*μ*g/mL) cells displayed very less or no effect at the same time. The aggressive effect of cisplatin on both cell lines was also examined. Plant extracts showed more cytotoxic effects on the viability of HepG2 cells at 400, 200, and 100 *μ*g/mL, whereas minimal effects were observed on normal cells (HEK293T). Results demonstrated that alcoholic extract had strong antiproliferative activity on cancer cells with a partial effect on HEK293T at 72 h, whereas, hexane extract showed negligible effects in all *in vitro* tested concentrations (10-400 *μ*g/mL).

### 3.2. Morphological Observation of Ethanolic Concentrations

Morphological assessment of ethanolic concentrations was observed in HepG2 and HEK293T cells shown in Figure 2. Alterations in cell structure, shape, and size were observed in a concentration-dependent manner. Cells at 50 *μ*g/mL and higher concentrations reduced the survival rate of cancer cells by losing their normal morphology and the capacity to attach to the surface. The lower concentration (10 *μ*g/mL) did not show any alteration in shape or reduced viability in HepG2 cells as observed by the MTT assay. In the case of cisplatin (positive control), a round-shaped image and less viability were observed in HepG2 treated cells. The morphological features and cytotoxicity of HEK293T cells were also assessed after treatment. Antiproliferative effects of ethanolic extract concentrations of *C. lindenii* stop the proliferation of cancerous cells, whereas healthy (HEK293T) cells were stable even at the highest concentration.

The article "In Vitro Evaluation of Cytotoxic Potential of Caladium lindenii Extracts on Human Hepatocarcinoma HepG2 and Normal HEK293T Cell Lines" was retracted in 2023. Reasons: signs of a paper mill; suspected computer-generated content; unreliable results or conclusions; concerns about the data.

### 3.3. Cell Viability Assay

Crystal violet staining is another way to assess the percentage viability of cells after treatment. The number of cells alive or adherent to the surface was estimated by using crystal violet staining of HepG2 and HEK293T cells as shown in Figure 3.

Effects of ethanolic and hexane extracts of *C. lindenii* on HepG2 cells with different concentrations starting from 10-400 *μ*g/mL showed different responses. Ethanolic concentrations showed a dose-depended decrease in percentage viability. HepG2 cells were exposed to ethanolic concentrations at 10, 50, 100, 200, and 400 *μ*g/mL found to be more toxic by measuring the absorbance at 570 nm. Staining facilitates the visualization of cell morphology by giving 100% of viability. Measurements were recorded as 78%, 67%, 50%, 37%, and 28% when treated with ethanolic concentrations exhibited a statistically significant decrease in HepG2 cells in comparison with negative control (99.5%). At higher concentrations of 200 and 400 *μ*g/mL, cell viability decreased to 37% and 28%, respectively. However, the viability assessment in healthy (HEK293T) cells were observed to be 95%, 90%, 88%, 76%, and 61% of ethanolic extract and 99% of DMSO. Upon treatment with hexane extracts showed 88%, 80%, 69%, 59%, 50% and 97% of DMSO cell viability. On the other hand, the nontumor HEK293T cells exhibited negligible effects on cell inhibition at 72 h with all concentrations of hexane extract. The observed cell viability of HEK293 treated cells was 97%, 95%, 88%, 75%, and 62%, and DMSO was 99.48%. Cisplatin concentration (10 *μ*g/mL) was administered to both cancer and healthy cells for the comparison of chemotherapeutic and natural antioxidants containing plant extracts. Percentage cell viability on HepG2 cells was 42%, while HEK293T exhibited 45% (Figure 3). R^2^ represents the coefficient of determination. Higher R-squared values demonstrate smaller differences between observed data and fitted values. Our results revealed a significant positive correlation (R^2^ = 0.9578, 0.9992, 0.9903, and 0.9885, *p* value<0.05) for both *C. lindenii* extracts.

### 3.4. Morphological Observation of Hexane Concentrations

The morphological observation showed the effect of hexane extract of *C. lindenii* on both HepG2 and HEK293T cells in Figure 4. *In vitro* treatment of hexane extract on HepG2 cells demonstrated mild alteration in cell morphology at all concentrations except the higher concentrations (200 and 400 *μ*g/mL). Cells treated with high concentrations of 200 and 400 *μ*g/mL became degraded and shrunken, while the lower concentrations of 10, 50, and 100 *μ*g/mL did not show satisfactory results. About 50% of cell reduction was calculated by percentage viability assay at 400 *μ*g/mL. The nontumor HEK293T cells showed normal morphology at all concentrations and did not show any sign of toxicity. Cisplatin (positive control) applied on healthy as well as cancer cells was observed with 45% and 42% of cell viability, respectively.

The article "In Vitro Evaluation of Cytotoxic Potential of Caladium lindenii Extracts on Human Hepatocarcinoma HepG2 and Normal HEK293T Cell Lines" was retracted in 2023. Reasons: signs of a paper mill; suspected computer-generated content; unreliable results or conclusions; concerns about the data.

## 4. Discussion

Modern technologies have underlined bioactive compounds and their importance in the world of drug discovery. A strong affiliation between flavonoids and anticancer activity has been reported in many studies [17]. Numerous active drugs are the byproduct of natural sources and are designed by the summation of synthetic polymers to overcome the burden of diseases [18]. Earlier researchers have demonstrated the phytochemical composition, antiproliferative, and antimicrobial potential of various *Caladium* species. Numerous studies have reported the antiangiogenic activity of methanolic extract of *C. bicolor* by inhibiting vascular endothelial growth factor (VEGF) signaling, a glycoprotein that promotes angiogenesis and vascular permeability. By this means, certain properties displayed are observed for the reduction of cancer growth and metastasis [19]. In Brazil, *C. lindenii* was used for the treatment of stingray wounds and other pathogenic infections. There is no pharmacological or phytochemical research has been reported on *C. lindenii*^12^.

Cell-based assays are used to determine the effect of compounds on cell growth or to monitor cytotoxic effects that ultimately lead to cell death. Despite prevailing circumstances of the cell-based assay, it is much more important to understand the remaining population of cells at the end of the reaction. MTT assay is the simplest and most effective method developed by Mosmann for quantifying *in vitro* chemo-sensitivity of applied drugs on human cancer cell lines. The principle of MTT assay is determined by the tetrazolium salt reduced into formazan crystals by the action of mitochondrial dehydrogenase enzyme that assists this function in living cells [20]. In this study, both extracts showed remarkably significant antiproliferative effects on the HepG2 cancer cell line, however, any sign of toxicity has not been observed in HEK293T cells. Calculated IC50 values for ethanolic and hexane extracts were assessed by MTT assay using different concentrations, i.e., 10, 50, 100, 200, and 400 *μ*g/mL showed that the ethanolic concentrations have high antiproliferative activity against HepG2 cells with IC50 = 31*μ*g/mL, while HEK293T cells exhibited minimal cytotoxicity even at the highest concentration with IC50 = 241*μ*g/mL. Hexane extract showed less cytotoxic effects on HepG2 (IC50 = 150*μ*g/mL) and statistically insignificant effects were found on normal human embryonic kidney cells with calculated IC50 = 550*μ*g/mL (Figure 1). The present study also demonstrated the sensitivity of liver cancer (HepG2) and normal (HEK293T) cells against an apoptosis-inducing agent (cisplatin). Cisplatin is an inorganic compound used for the treatment of various malignancies including gastric, bladder, and prostate cancer by inhibiting the DNA replication and transcription events. The severe side effects of cisplatin as an anticancer drug also triggered drug resistance and the termination of normal cell proliferation by damaging DNA [21]. However, the potential organic extracts were more effective against HepG2 cells as compared to HEK293T cells with favorable IC50 values. In this study, cisplatin showed an anticancer effect on HepG2 and an adverse effect on the normal morphology of HEK293T cells when compared with UT (untreated) and DMSO (negative control) (Figures 2, 4). Cancer cells are categorized and recognized from normal cells due to their high proliferative and colony-forming potential. Drug discovery involves a complex mechanism that demands the assessment of the cell viability of living cells on cultured cancer and normal cells. Crystal violet is the simple method to calculate the sustained cells with crystal violet staining dye that binds to DNA and proteins. During the assay, the dead cells were detached from the surface and vanished from the cell population. This practice describes a standard outline for the analysis of plant extracts on cell survival and growth inhibition [22]. In this study, cell viability was calculated using crystal violet staining of HepG2 and HEK293T cells as described in Figure 3 and Table 2 as mean ± SD. The cell population was measured for two cell lines by obtaining optical densities and plotting a curve and slope. It has been observed that drug response is directly proportional to cell density in a time-dependent manner. The decreased percentage signifies strong cytotoxicity of plant extracts against hepatocellular carcinoma, whereas an increased value showed less effect on dose concentration. The percentage viability of ethanolic concentrations (10, 50, 100, 200, and 400 *μ*g/mL) decreases with the increase in dose. The higher concentrations of 200 and 400 *μ*g/mL showed reduced percentage viability on calculation. While evaluating hexane extract, the cell viability displayed more viable cells indicating less cytotoxicity on HepG2 cells, otherwise, HEK293T cells showed increased cell viability with minimal or no effects. The microscopic assessment revealed a clear dose-dependent decrease in cell density and altered morphology of HepG2 cells with ethanolic and *n*-hexane extract concentrations.

The article "In Vitro Evaluation of Cytotoxic Potential of Caladium lindenii Extracts on Human Hepatocarcinoma HepG2 and Normal HEK293T Cell Lines" was retracted in 2023. Reasons: signs of a paper mill; suspected computer-generated content; unreliable results or conclusions; concerns about the data.

## 5. Conclusion

The crude organic extracts of *C. lindenii* showed remarkable cytotoxicity against the HepG2 cell line by inducing apoptosis and significantly reducing viability percentage and transforming morphology in a dose-dependent manner. The activity exhibited by ethanolic extract showed the most favorable results for HepG2 cells as compared to hexane extract. However, these extracts show minimal or no effects on the healthy HEK293 cell line. These findings justify the antiproliferative activity of *C. lindenii* that may be used for the specific treatment of cancer after further validations.

## Figures and Tables

**Figure 1:** Graphical representation: *In vitro* assessment of ethanolic and hexane extracts of *C. lindenii* on HepG2 and HEK293T cell lines. (a) MTT assay results showed a significantly increased mortality rate of HepG2 cells after treatment with higher concentrations at 72 h. (b) HEK293T being a normal cell line revealed less toxicity of ethanolic extract only at the highest concentrations (400, 200 *μ*g/mL) as compared to hexane extract. (c) Hexane concentration on HepG2 cells showed less effect. (d) HEK293T cell line revealed less or no activity of hexane extract. Cisplatin was used as positive control and showed more negative effects against normal cell line, however, DMSO was taken as a negative control. ^∗^*p*˂0.05, ^∗∗^*p*˂0.001, and ^∗∗∗^*p*˂0.0001 referred as statistically significant. Error bars showed error or standard deviation as mean ± SD of each group. MTT: 3-(4, 5-dimethylthiazol-2yl)-2, 5-biphenyl tetrazolium bromide; DMSO: dimethyl sulfoxide; SD: standard deviation.

**Figure 2:** Morphological representation of HepG2 cells following the exposure of increasing concentrations of ethanolic extract of *C. lindenii* at 72 h observed by Floid cell imaging station. Changes in the morphology of hepatocellular carcinoma (HepG2) cells are very obvious when exposed to ethanolic concentrations. (a) The concentration of 50 *μ*g/mL and higher changed the normal morphology and the cell adhesion capability to the surface as compared to the control. Higher cellular concentrations give the impression of clusters. The lower concentration (10 *μ*g/mL) did not show altered shape or reduced viability in HepG2 cells as observed by the MTT assay. Application of cisplatin (positive control) changed the morphology of both cancerous and healthy cells round-shaped with less viability. (b) The morphological features and cytotoxicity of *C. lindenii* on normal cells (HEK293T) did not show a negative effect even at the highest concentration. However, the drug (cisplatin) response elaborated altered cellular morphology. MTT: 3-(4,5-dimethylthiazol-2yl)-2,5-biphenyl tetrazolium bromide; DMSO: dimethyl sulfoxide.

The article "In Vitro Evaluation of Cytotoxic Potential of Caladium lindenii Extracts on Human Hepatocarcinoma HepG2 and Normal HEK293T Cell Lines" was retracted in 2023. Reasons: signs of a paper mill; suspected computer-generated content; unreliable results or conclusions; concerns about the data.

**Figure 3:** The growth rate of cells was calculated by the crystal violet staining protocol. Optical density (OD) at 570 nm was measured and plotted to obtain the percentage viability of untreated, treated, and control cells. In cell viability assay, a drug response is driven by cell density. A trend-line slope showed the number of cells/well certified to be significant. (a) The calculated percentage elaborated a clear dose-dependent decrease in HepG2 cells with significant R^2^ (coefficient of determination) values. (b) HEK293T plotted slope remained constant with a slight fall and showed good viability. (c) Hexane extract showed 59% and 50% viability on HepG2 cells at higher (200 and 400 *μ*g/mL) concentrations. (d) Nontumor cells did not show the activity of hexane extract at any concentration. Statistical analysis described as ^∗^*p*˂0.05, ^∗∗^*p*˂0.001, and ^∗∗∗^*p*˂0.0001. DMSO: Dimethyl sulfoxide; SD: standard deviation; CV: crystal violet; MTT: 3-(4, 5-dimethylthiazol-2yl)-2, 5-biphenyl tetrazolium bromide.

**Figure 4:** The morphological features showed the effect of hexane extract of *C. lindenii* on both HepG2 and HEK293T cells. (a) *In vitro* treatment of hexane extract on HepG2 cells demonstrated mild alteration in cell morphology at all concentrations except the higher (200 and 400 *μ*g/mL) concentrations. The lower concentrations 10, 50, and 100 *μ*g/mL did not show satisfactory results. Cells treated with high concentrations became degraded and shrunken. 50% of cell reduction was calculated by percentage viability assay at 400 *μ*g/mL. (b) The nontumor HEK293T cells showed normal morphology at all concentrations and did not reveal any sign of toxicity in comparison with UT and DMSO (negative control). Cisplatin (10 *μ*g/mL) was the positive control applied on healthy (HEK293T) as well as cancer (HepG2) cells showed 45% and 42% of cell viability, respectively.

**Table 1:** MTT assay results.

Cell lines	Absorbance (at 570 nm) mean ± SD								
	Solvents	UT	DMSO	10 *μ*g/mL	50 *μ*g/mL	100 *μ*g/mL	200 *μ*g/mL	400 *μ*g/mL	Cisplatin 10 *μ*g/mL
HepG2	Ethanol	0.0661 ± 0.0018	0.0653 ± 0.0015	0.0434 ± 0.0079	0.0284 ± 0.00043	0.022 ± 0.0011	0.0157 ± 0.0019	0.011 ± 0.001	0.0417 ± 0.0042
	Hexane	0.0662 ± 0.00015	0.0655 ± 0.00066	0.0611 ± 0.000346	0.0523 ± 0.00211	0.0413 ± 0.00125	0.0313 ± 0.00153	0.0215 ± 0.00052	0.0386 ± 0.00390
HEK293T	Ethanol	1.8313 ± 0.0107	1.8115 ± 0.00908	1.7544 ± 0.05288	1.5735 ± 0.00083	1.4017 ± 0.00971	1.1199 ± 0.0379	0.8477 ± 0.0642	0.7534 ± 0.0146
	Hexane	1.8937 ± 0.05147	1.9543 ± 0.0330	1.9662 ± 0.02862	1.7962 ± 0.04726	1.6266 ± 0.02160	1.4058 ± 0.07346	1.1541 ± 0.01872	0.8273 ± 0.08484

The article "In Vitro Evaluation of Cytotoxic Potential of Caladium lindenii Extracts on Human Hepatocarcinoma HepG2 and Normal HEK293T Cell Lines" was retracted in 2023. Reasons: signs of a paper mill; suspected computer-generated content; unreliable results or conclusions; concerns about the data.

**Table 2:** Crystal violet assay results.

Cell lines	Absorbance (at 570 nm) mean ± SD								
	Solvents	UT	DMSO	10 *μ*g/mL	50 *μ*g/mL	100 *μ*g/mL	200 *μ*g/mL	400 *μ*g/mL	Cisplatin 10 *μ*g/mL
HepG2	Ethanol	0.0647 ± 0.00062	0.0613 ± 0.00055	0.0518 ± 0.0013	0.0403 ± 0.0029	0.0304 ± 0.00043	0.0217 ± 0.00078	0.0127 ± 0.0011	0.0333 ± 0.00179
	Hexane	0.0659 ± 0.0021	0.0652 ± 0.00198	0.0554 ± 0.00671	0.0522 ± 0.000141	0.0450 ± 0.00091	0.0382 ± 0.00021	0.0320 ± 0.0044	0.0321 ± 0.00023
HEK293T	Ethanol	1.8457 ± 0.0128	1.8362 ± 0.00513	1.7355 ± 0.01655	1.5355 ± 0.01022	1.4368 ± 0.00804	1.2061 ± 0.05218	0.9512 ± 0.00438	0.6628 ± 0.02832
	Hexane	1.9427 ± 0.01682	1.8898 ± 0.05844	1.8996 ± 0.06039	1.7944 ± 0.05833	1.6735 ± 0.05427	1.4245 ± 0.02889	1.1615 ± 0.01011	0.8154 ± 0.1153

## Data Availability

All datasets used and analyzed during the current study are available from the corresponding author on reasonable request.

## References

[1] Garcia-Oliveira P., Otero P., Pereira A. G. (2021). Status and challenges of plant-anticancer compounds in cancer treatment. *Pharmaceuticals.*.

[2] Sung H., Ferlay J., Siegel R. L. (2021). Global cancer statistics 2020: GLOBOCAN estimates of incidence and mortality worldwide for 36 cancers in 185 countries. *CA: a Cancer Journal for Clinicians*.

[3] Emam M. A., Khattab H. I., Hegazy M. G. (2019). Assessment of anticancer activity ofPulicaria undulataon hepatocellular carcinoma HepG2 cell line. *Tumor Biology*.

[4] Mirabelli P., Coppola L., Salvatore M. (2019). Cancer cell lines are useful model systems for medical research. *Cancers*.

[5] Dagogo-Jack I., Shaw A. T. (2018). Tumour heterogeneity and resistance to cancer therapies. *Nature Reviews Clinical Oncology*.

[6] Santos-Sánchez N. F., Salas-Coronado R., Hernández-Carlos B., Villanueva-Cañongo C. (2019). Shikimic acid pathway in biosynthesis of phenolic compounds. *Plant physiological aspects of phenolic compounds*.

[7] Pinto T., Aires A., Cosme F. (2021). Bioactive (poly) phenols, volatile compounds from vegetables, medicinal and aromatic plants. *Food*.

[8] Bisht R., Bhattacharyya A., Shrivastava A., Saxena P. (2021). An overview of the medicinally important plant type III PKS derived polyketides. *Frontiers in Plant Science*.

The article "In Vitro Evaluation of Cytotoxic Potential of Caladium lindenii Extracts on Human Hepatocarcinoma HepG2 and Normal HEK293T Cell Lines" was retracted in 2023. Reasons: signs of a paper mill; suspected computer-generated content; unreliable results or conclusions; concerns about the data.

[9] Newman D. J., Cragg G. M. (2016). Natural products as sources of new drugs from 1981 to 2014. *Journal of Natural Products*.

[10] Roy A., Bharadvaja N. (2017). Medicinal plants in the management of cancer: a review. *Int J Complement Alt Med.*.

[11] Uche F. I., Onuchukwu D., Ibezim C. N. E., Ogbu H. I. (2019). Methanolic extract of Caladium bicolor leaves against selected clinical isolates. *GSC biol. pharm. sci.*.

[12] Zhang D., Arunachalam K., Wang Y. (2021). Evaluation on antidiabetic properties of medicinal plants from Myanmar. *Scientific World Journal*.

[13] Mukavi J. W., Mayeku P. W., Nyaga J. M., Kituyi S. N. (2020). In vitro anti-cancer efficacy and phyto-chemical screening of solvent extracts of Kigelia africana (Lam.) Benth. *Heliyon*.

[14] Masuku N. P., Lebelo S. L. (2019). Investigation of the effects of Kigelia africana (Lam.) Benth. Extracts on TM3 Leydig cells. *Asian Journal of Pharmaceutical and Clinical Research*.

[15] Riaz S., Javed M. A., Nawaz I., Javed T. (2022). Biochemical characterization, cytotoxic, antimutagenic, anticancer and molecular docking studies on Tecomella undulata. *Saudi J. Biol. Sci.*.

[16] Nawaz A., Jamal A., Arif A., Parveen Z. (2021). In vitro cytotoxic potential of _Solanum nigrum_ against human cancer cell lines. *Saudi J. Biol. Sci.*.

[17] Muthuvel A., Jothibas M., Manoharan C. (2020). Effect of chemically synthesis compared to biosynthesized ZnO-NPs using _Solanum nigrum_ leaf extract and their photocatalytic, antibacterial and in- vitro antioxidant activity. *Journal of Environmental Chemical Engineering*.

[18] Lelario F., Scrano L., De Franchi S. (2018). Identification and antimicrobial activity of most representative secondary metabolites from different plant species. *Chemical and Biological Technologies in Agriculture*.

[19] Tosoc J. P., Frediles V. C., Canda C., Demayo C. G. (2016). Antiangiogenic, antitoxic and antioxidant properties of methanolic extracts of Caladium bicolor (Aiton) Venten. *Human and Veterinary Medicine*.

[20] Kamiloglu S., Sari G., Ozdal T., Capanoglu E. (2020). Guidelines for cell viability assays. *Food Frontiers.*.

[21] Qi L., Luo Q., Zhang Y., Jia F., Zhao Y., Wang F. (2019). Advances in toxicological research of the anticancer drug cisplatin. *Chemical Research in Toxicology*.

[22] Garg S., Huifu H., Kaul S. C., Wadhwa R. (2018). Integration of conventional cell viability assays for reliable and reproducible read-outs: experimental evidence. *BMC Research Notes*.

